# Case report: locoregional (perineum and inguinal) recurrence after treatment of rectal cancer by low anterior resection

**DOI:** 10.1186/1477-7819-11-186

**Published:** 2013-08-12

**Authors:** Rong Zhao, Li Zhang

**Affiliations:** 1 Department of Colorectal Surgery, Tianjin Union Medicine Center, 190 Jieyuan Road, Hongqiao District, 300121 Tianjin, China; 2 Department of Pathology, Tianjin Union Medicine Center, 190 Jieyuan Road, Hongqiao District, 300121 Tianjin, China

**Keywords:** Local recurrence, Rectal cancer resection, Pathology analysis, Adenocarcinoma

## Abstract

This report presents a case of perineal and inguinal recurrence and metastasis after treatment of rectal cancer by low anterior resection. A 57-year-old Chinese woman was diagnosed with rectal cancer in September 2008. The tumor and metastasis were recurrent many times in the perineum and inguinal regions from first diagnosis to October 2011. Twelve surgeries were performed and several nodules were removed. Adjuvant radiation therapy and chemotherapy were also carried out. Pathological analysis indicated that most nodules were adenocarcinoma. The interesting finding was that this case did not seem to belong to any traditional rectal cancer metastasis pathway. This case is representative and worthy of further study to explore whether there is another rectal cancer metastasis pathway.

## Background

Local recurrence (LR) of rectal cancer is defined as an occurrence of the recurrent disease in the pelvis after a surgical resection. However, inguinal lymph nodes do not belong to the regional lymph nodes of rectal cancers according to the Union for International Cancer Control (UICC) TNM staging classification. Generally, inguinal lymph node metastasis is not included in LR of rectal cancers [1]. LR after a rectal resection can cause high morbidity and can severely lower quality of life [1-5].

More than 50% of LRs of rectal cancer are independent occurrence cases and many patients (30% to 50%) are reported to die without evidence of distant metastases [6]. In most cases, 55% to 80% of LRs occur in the second year after the operation and rarely occur beyond 5 years [7]. There appears to be a significant correlation between LR rates and survival rates, with high LR rates reducing survival rates.

Although autopsy studies have suggested that patients may die from disseminated reoccurrence without symptoms, all LRs eventually cause symptoms such as pelvic and/or perianal pain or rectal bleeding [8,9]. For some patients, the carcinoembryonic antigen (CEA) is a biomarker for LR, but the role of CEA in follow-up is still debated. Any additional useful information is not offered by other serum markers.

Three points need to be addressed: first, which biomarkers and indices are beneficial in routine follow-up after a curative (R0) resection for patients with rectal cancer, including CEA; second, if LR is suspected, which method provides the best diagnostic accuracy; and third, how to classify the stage of LR with the aim of further surgical resection. Even with close surveillance, more than half of patients would be diagnosed with LR after onset of symptoms such as perineum, low back or pelvic pain. Routine follow-up may identify recurrences at an earlier stage and many methods can be conducted for treatment [10-12].

Most patients with LRs have advanced local and/or disseminated disease at the time of diagnosis. The LC can be found by imaging modalities such as magnetic resonance imaging (MRI), computed tomography (CT) and positron emission tomography - computed tomography (PET-CT), and further confirmed by biopsy. A number of studies have demonstrated that some LRs can be resected with curative intent and long-term survival can be achieved in a few patients [13,14]. Usually, further radiotherapy can be given to patients based on previous history of radiotherapy and dosage received, as this is a multidisciplinary decision [15,16], whereas the use of adjuvant chemoradiation is based on clinical evidence. The minimum resection margin has not been well defined. A previous study suggested that a palliative resection (R1 to R2) of the LR is unlikely to benefit the majority of patients [17]. Symptomatic patients might be offered radiotherapy, otherwise treatment depends on the burden of disease and whether it is only local or disseminated; a complex issue that needs to be addressed at multidisciplinary level. Chemotherapy should be recommended to patients with severe metastatic conditions [9].

## Case presentation

A 57-year-old Chinese woman presented to Tianjin Union Medicine Center, Tianjin, China, with rectal adenocarcinoma at Dukes’ stage C. Before presenting to the hospital, the patient was not taking any drugs and had a completely negative medical history. On 7 October 2008, the patient was treated by low anterior resection, at a distance of 13 cm from the anus and radical resection was performed. Before surgery, it was not known whether the patient had lymph node metastasis or whether the tumor, which was not large in size, could be completely resected by surgery, and so neoadjuvant chemoradiotherapy was not performed.

Following the operation, from 31 October 2008 to 10 April 2009, chemotherapy treatment (oxaliplatin) was carried out five times every month with a total of six cycles. On 4 June 2009, six lesions with a maximum diameter of 0.5 cm were removed by inner lens polyp resection. Six months later, a lesion measuring 2.3 cm × 1.4 cm, at a distance of 0.5 cm from the left side of perianal region, was removed and pathology analysis indicated adenocarcinoma. On 13 March 2010, another lesion measuring 1.5 cm × 1.0 cm × 1.0 cm was removed from the left groin. Pathology analysis indicated lymph node metastasis. Figure 1a shows the pathological findings of this lesion. On 31 March 2010, the patient could not tolerate chemotherapy with irinotecan and so chemotherapy was terminated. From 12 April 2010 to 18 June 2010, the patient received radiation therapy on the bilateral inguinal region and anus 32 times, including 10 times with enhanced radiation therapy. On 6 August 2010, a perianal lesion measuring approximately 1.3 cm × 0.8 cm × 0.9 cm, 1 cm from the left anterior anal wall (close to the perineum), was removed. Pathology analysis indicated adenocarcinoma with cytokeratin CK20^+^ (Figure 1b). There was a small postoperative anal defect in the patient. On 30 September 2010, multiple right inguinal nodules, measuring a maximum of approximately 1.6 cm × 0.7 cm, were removed. Pathology analysis indicated metastatic lymph node adenocarcinoma (5/7 nodules). On 11 November 2010, the perianal nodules (measuring 2.2 cm × 1.3 cm × 0.3 cm), the adenocarcinoma nodules in the skin and subcutaneous tissue, and three right inguinal nodules (CK^−^) (measuring a maximum 1.4 cm × 1.4 cm), were resected (Figure 1c).

**Figure 1:** **Pathological findings of patient in 2010. (a)** On 13 March 2010, a lesion was removed from the left groin and pathology indicated lymph node metastasis. **(b)** On 6 August 2010, a perianal lesion from the left anterior anal wall was removed and pathology indicated adenocarcinoma (CK20^+^). **(c)** On 11 November 2010, perianal tumors were resected (CK^+^, CEA^+−^). CEA, carcinoembryonic antigen; CK, cytokeratin.

On 23 February 2011, three perianal tumors (measuring 2.0 cm × 2.0 cm × 0.4 cm; CK^+^, CEA^+−^), 0.3 cm to 1.3 cm from the anal margin and left posterior anal wall of the external sphincter (left, middle and rear), were resected (Figure 2a). On 31 May 2011, the left inguinal lymph node was resected and analysis indicated lymphadenia (measuring 1.0 cm × 1.5 cm × 0.2 cm) (Figure 2b). The anal margin tumor near the location of the nodule, found on 6 August 2010, was resected and pathology analysis indicated adenocarcinoma (measuring approximately 0.6 cm × 0.7 cm × 0.2 cm). On 23 September 2011, tissue measuring 0.9 cm × 0.5 cm × 0.7 cm was removed, but analysis indicated that it was adipose tissue. On 25 October 2011, the perianal lesions (measuring 1.4 cm × 0.6 cm × 0.8 cm; near the last end tailbone) left behind the anal margin were removed. Pathology analysis indicated CK staining was negative (Figure 2c).

**Figure 2:** **Pathological findings of patient in 2011. (a)** On 23 February 2011, tumors from the anal margin and left posterior anal wall of the external sphincter were resected (CK^+^, CEA^+−^). **(b)** On 31 May 2011, the left inguinal lymph node was resected and analysis indicated lymphadenia. **(c)** On 25 October 2011, perianal lesions left behind the anal margin were removed (CK^−^). CEA, carcinoembryonic antigen; CK, cytokeratin.

Following the initial resection surgery, the patient attended hospital for surveillance examination every 3 months. B-mode ultrasonography, chest X-ray and blood biomarker tests were performed. Every 6 months, CT scanning was used to find any LR and distant metastasis. Until 9 April 2013, the patient is alive and has good condition.

## Conclusions

We reported this case for several reasons. First, the case presented a rare clinicopathological condition, which was unusual because of the low incidence of LR and the quantity of surgeries undertaken. Generally, LR rates can be related to the surgeon’s skill and experience. LR rates can be approximately halved by adjuvant radiation therapy (pre- or postoperatively, with or without supplementary chemotherapy) or by optimization of the surgical technique [18]. Second, this patient was treated with surgery, adjuvant radiation therapy and chemotherapy, which are almost all routine methods for rectal cancer and locoregional recurrence [16]. Currently, there are three principal surgical methods: Hartmann’s procedure (for patients with LR after a previous anterior resection), pelvic exenteration and abdominosacral resection. The type of operation must be tailored to each patient and no general rule can be given [12-15]. Based on the published literature and beneficial effects of adjuvant radiation therapy on patients with primary local rectal cancer, there is consensus that radiation therapy should be carried out on all patients receiving surgical resection for LR. However, there is no evidence based on specifically designed and analyzed studies to suggest that chemotherapy can add benefit to patients with independent LR. There is also no evidence that immunotherapy using interferon or other immune drugs improves outcomes.

Generally, the rectal cancer metastasis pathway includes blood spread, lymphatic spread, direct spread and planting [19]. An interesting observation was that this case was unlikely to belong to any of these pathways. The blood drainage area of rectal cancer was the liver and lung through blood circulation. The lymphatic drainage area of the rectal cancer was rare to include the groin, only noted in about 2.5% of patients [20]. Direct spread and planting do not seem to reach the LR area in this case either, because of the pelvic diaphragm (including the portion of the pelvic floor formed by the coccygeal and levator ani muscles, and their fasciae) between the rectum and anus, and it is difficult to reach the LR by direct spread and planting. We did not find any lesions and metastasis on the tissues of the pelvic diaphragm. In general, cutaneous and subcutaneous recurrence occurs after lung and liver metastasis. However, we did not find any organ metastasis occurrence, including the lungs, liver and brain, even by PET-CT examination. Therefore, this case was representative, since it does not belong to any traditional rectal cancer spread pathway and is worthy of further study to explore whether there is another rectal cancer metastasis pathway.

## Consent

The patient gave written informed consent for this case report to be published.

## Abbreviations

CEA: carcinoembryonic antigen; CK: cytokeratin; CT: computed tomography; LR: local recurrence; MRI: magnetic resonance imaging; PET-CT: positron emission tomography - computed tomography; UICC: Union for International Cancer Control.

## Competing interests

The author declares no conflicts of interest.
